The article "Long Noncoding RNA UCA1 Regulates PRL-3 Expression by Sponging MicroRNA-495 to Promote the Progression of Gastric Cancer" was retracted in 2022. Reasons: manipulated images; duplicated images.

# Long Noncoding RNA UCA1 Regulates PRL-3 Expression by Sponging MicroRNA-495 to Promote the Progression of Gastric Cancer

**DOI:** 10.1016/j.omtn.2019.10.020

**Published:** 2019-10-25

**Authors:** Yi Cao, Jian-Bo Xiong, Guo-Yang Zhang, Yi Liu, Zhi-Gang Jie, Zheng-Rong Li

**Affiliations:** 1 Department of Gastroenterological Surgery, The First Affiliated Hospital of Nanchang University, Nanchang 330006, P.R. China

**Keywords:** long noncoding RNA UCA1, microRNA-495, PRL-3, gastric cancer

## Abstract

Gastric cancer (GC) is among the most frequently occurring malignancies worldwide. In recent years, long noncoding RNAs (lncRNAs) have been widely studied because of their ability to regulate the cellular processes involved with tumorigenesis. The present study aims to investigate the underlying molecular mechanism by which lncRNA urothelial carcinoma-associated 1 (UCA1) influences the progression of GC. Differentially expressed lncRNA UCA1 was initially identified by microarray-based analysis, after which a high expression of UCA1 was determined in GC tissues and cells. It is important to note that UCA1 could upregulate the expression of phosphatase of regenerating liver-3 (PRL-3) by sponging miR-495. The expression of UCA1 and miR-495 was altered in human GC cells to evaluate cell activity *in vitro*, as well as peritoneal metastasis and tumor formation ability *in vivo*. Results suggested that increased expression of UCA1 promoted cell proliferation, migration, and invasion, accompanied by suppressed cell apoptosis, as well as enhanced peritoneal metastasis and tumorigenesis of GC cells. Meanwhile, the upregulated expression of miR-495 could reverse the promotive effects exerted by UCA1. Taken conjointly, UCA1, as a competing endogenous RNA (ceRNA) of miR-495, could accelerate the development of GC by upregulating PRL-3, highlighting a potentially promising basis for the targeted intervention treatment of GC.

## Introduction

Gastric cancer (GC) is a severe public health burden, leading to over 723,000 deaths worldwide on an annual basis.^1^^,^^2^ The incidence of GC follows a wide geographical variation, where Asian countries including China, Japan, and Korea exhibit the highest incidence rate of GC in comparison with the rest of the world.^3^ Risk factors contributing to the incidence of GC include *Helicobacter pylori* infection, dietary habits, tobacco use, and obesity.^4^ Although the incidence and mortality rates of GC have declined in recent years, it still represents one of the leading causes of cancer-related deaths worldwide.^5^ At present, surgical resection of the stomach with lymph node dissection represents the most effective therapeutic approach for GC. However, the prognosis and survival of advanced GC remain poor.^6^ Tumor invasion and metastasis are two crucial factors contributing to poor prognosis in patients suffering from cancer. Almost 80% of GC recurrences present as peritoneal metastasis, with the underlying mechanism continuing to elude researchers and clinicians alike.^7^ Recent studies have uncovered promising possible cellular targets for drug treatment; however, current molecular biology and advanced treatment options of GC still require further analysis and better understanding.^8^, ^9^, ^10^

Long noncoding RNAs (lncRNAs) are a class of RNAs comprised of 200 nucleotides or more, with little or no protein-coding potential.^11^^,^^12^ Previous studies have highlighted the importance and ability of lncRNAs in their involvement in various biological progresses of malignancies including proliferation, differentiation, and metabolism.^13^ In addition, lncRNAs are versatile in regulating capabilities where they are able to modulate both transcriptional and the post-transcriptional processes.^14^ Located on human 19p13.12, urothelial carcinoma-associated 1 (UCA1) is a member of lncRNA with three exons.^15^ UCA1 overexpression has been previously demonstrated to play a role in various cancer types including GC, non-small cell lung cancer, bladder carcinoma, tongue squamous cell carcinoma, ovarian cancer, esophageal squamous cell carcinoma, and hepatocellular carcinoma.^16^^,^^17^ Based on the current existing literature, UCA1 is able to function as an oncogenic lncRNA in various types of cancers, which makes it a suitable target molecule to study.

MicroRNAs (miRNAs) are noncoding RNAs 20–24 nt in length that are capable of modulating stability and translational efficiency of target mRNAs.^18^ miRNAs regulate various biological processes such as cellular proliferation, cell differentiation, metabolic signaling, and apoptosis.^19^ The differential expression of miRNAs between normal and cancer tissues has been extensively studied in a diverse range of cancers, all of which highlight a relationship between miRNA expression and cancer progression.^20^ In GC, the miR-106b-25 cluster has been shown to be involved in E2F1 post-transcriptional regulation, as well as having an effect on transforming growth factor β (TGF-β) resistance development.^21^ As demonstrated by another example, miR-375 was found to regulate cell proliferation and suppress tumor growth by targeting the JAK2 oncogene.^22^ Studies have shown how deregulated miRNAs could act as tumor suppressors or oncogenes correspondingly, and with this in mind, we subsequently proposed that the deregulation of a candidate miRNA, namely, miR-495, could potentially be a mechanism in triggering the downregulation of tumor suppressors in tumors.

Phosphatase of regenerating liver-3 (PRL-3) encodes a 22-kDa protein that represents a member of a superfamily of protein tyrosine phosphatases (PTPs) that are ubiquitously expressed in a host of tumors. The PRL-PTP family is composed of three members, PRL-1, PRL-2, and PRL-3.^23^ Saha et al.^24^ demonstrated that PRL-3 acted as a metastasis-related gene that was increased in metastatic colorectal cancer. Furthermore, PRL expression (particularly the expression of PRL-3) has been demonstrated to share an association with cellular motility, invasion, and metastasis in various types of tumors, including that of GC, ovarian cancer, colorectal cancer, breast cancer, and lung cancer.^25^

With increased understanding of the aforementioned factors and the potential molecular mechanisms involved in GC, we designed a series of *in vivo* and *in vitro* experiments aimed at investigating the underlying relationships of UCA1, PRL-3, and miR-495 in GC cells in hopes of uncovering a novel therapeutic target in the treatment of GC.

## Results

### UCA1 Was Highly Expressed in GC Tissues and Cell Lines

GEO: GSE65801 and GSE103236 microarray data showed that UCA1 was upregulated in GC (Figures 1A and 1B). qRT-PCR results indicated that the relative expression of UCA1 was higher in GC tissues than that of their comparative adjacent normal tissues (Figure 1C), with higher expression recorded in GC cells (MKN-28, MKN-45, SGC-7901, BGC-823, and MGC-803) than in normal gastric epithelial cells (GSE-1) (Figure 1D) (all p < 0.05). Based on the obtained data, the BGC-823 cell line with highest expression of UCA1 was selected for further experiments. According to the mean expression of UCA1, the UCA1 expression of samples was assigned into low UCA1 expression and high UCA1 expression. Kaplan-Meier method with log rank test was used to analyze the relationship between UCA1 expression and GC patient survival, and the results showed that GC patients with low expression of UCA1 were observed with prolonged survival (p < 0.05) (Figure 1E). We further analyzed the relationship between the UCA1 expression and the clinicopathological characteristics observed among GC patients. Results (Table S1) showed that expression levels of UCA1 were not related to factors of gender, age, tumor site, and tumor size of patients. However, a strong correlation was observed between clinical stage, lymph node metastasis, and tumor infiltration depth.

**Figure 1:** UCA1 Was Highly Expressed in GC Tissues and GC Cells (MKN-28, MKN-45, SGC-7901, BGC-823, and MGC-803) (A) Heatmap of GSE65801. *p < 0.05, versus the adjacent normal tissues. (B) Heatmap of GSE103236. The abscissa represents the sample number, the ordinate represents the differentially expressed gene name, the upper right histogram is the color order, the top-down color change represents the expression value of the chip data from large to small, each rectangle corresponds to the expression value of a sample, and each column represents the expression level of all genes in each sample. The left tree chart shows the clustering analysis results of different genes from different samples. The top bar indicates the type of sample, the upper right box indicates the color reference of the sample, the blue is the normal control sample, and the red is the tumor sample. (C) UCA1 was highly expressed in GC tissues (n = 85). (D) UCA1 was highly expressed in GC cells (MKN-28, MKN-45, SGC-7901, BGC-823, and MGC-803). *p < 0.05, versus the GSE-1 cell line; ^#^p < 0.01, versus the GSE-1 cell line. (E) Kaplan-Meier analysis shows that expression of UCA1 is negatively correlated with GC patient survival (the measurement data in GC cell lines were analyzed by one-way ANOVA, and the measurement data in GC and adjacent normal tissues were analyzed by paired t test, each experiment was conducted three times independently).

### UCA1 Was Mainly Located in the Cytoplasm of GC Cells

As illustrated in Figure 2, the online analysis software employed predicted that UCA1 was located in the cytoplasm of GC cells. RNA-fluorescence *in situ* hybridization (FISH) analysis further supports and verifies our findings.

**Figure 2:** UCA1 Is Mainly Localized in the Cytoplasm of GC Cells (A) Bioinformatics analysis predicted that UCA1 is located in the cytoplasm of GC cells. (B) FISH assay (original magnification ×400) verified that UCA1 is located in the cytoplasm of GC cells.

### UCA1 Is Upregulated PRL-3 by Sponging miR-495

Through prediction of the bioinformatics database microrna.org (http://www.microrna.org/microrna/getMirnaForm.do), we found that there were potential binding sites between UCA1 and miR-495. As the candidate miRNA of UCA1, miR-495 was screened using the bioinformatics website. We discovered that there was a specific binding point between miR-495 and UCA1 (Figure 3A). Dual-luciferase (Luc) reporter assay (Figure 3B) revealed that when co-transfected with UCA1-WT (wild-type)-Luc, the Luc activity of the miR-495 mimic group was significantly lower than that of the miR-495 mimic-negative control (NC) group (p < 0.05), whereas those co-transfected with UCA1-Mut (mutant)-Luc led to no significant changes in Luc activity in each group (p > 0.05). Additionally, target genes of miR-495 were predicted by TargetScan (http://www.targetscan.org/vert_71/), which suggested that the potential target gene for miR-495 was PRL-3 (Figure 3C). Dual-Luc reporter assay (Figure 3D) indicated that when co-transfected with PRL-3-WT-Luc, the Luc activity of the miR-495 mimic group was significantly lower in comparison with those in the miR-495 mimic-NC group (p < 0.05), whereas no significant differences were observed in the Luc activity in each group when co-transfected with PRL-3-Mut-Luc (p > 0.05). RNA pull-down results showed that UCA1 was significantly higher in WT-miR-495 when compared with Mut-miR-495 (p < 0.05), indicating that miR-495 was directly bound to UCA1 (Figure 3E). Results from RNA binding protein immunoprecipitation (RIP) assay reflect how UCA1 was significantly enriched within Ago2 when compared with immunoglobulin G (IgG) (p < 0.05), indicating that UCA1 was directly bound to Ago2 (Figure 3F).

**Figure 3:** UCA1 Competitively Binds to miR-495 to Upregulate PRL-3 (A) The targeting relationship between UCA1 and miR-495 predicted by the bioinformatics website. (B) The targeting relationship between UCA1 and miR-495 verified by dual-Luc reporter gene assay. (C) The targeting relationship between PRL-3 and miR-495 predicted by the bioinformatics website. (D) The targeting relationship between PRL-3 and miR-495 verified by dual-Luc reporter gene assay. (E) miR-495 binds to UCA1 by RNA pull-down assessment. (F) miR-495 binds to UCA1 by RIP assay. (G) miR-495 was negatively correlated with UCA1. (H) PRL-3 was negatively correlated with miR-495. (I) Expressions of UCA1, miR-495, and PRL-3 detected by qRT-PCR in each group. *p < 0.05, versus the other three groups in (B) and (E), versus the Bio-NC probe-labeled group in (C), versus the IgG group in (F), and versus the control group in (G) (comparisons between two groups were made using paired t test; comparisons of measurement data among multiple groups were analyzed by one-way ANOVA; each experiment was conducted three times independently).

qRT-PCR was used to detect the UCA1, miR-495, and PRL-3 expression in GC tissues, and analyze their correlation. The results showed that miR-495 expression was negatively correlated with UCA1 expression (Figure 3G), and PRL-3 expression was also negatively correlated with miR-495 (Figure 3H). Furthermore, qRT-PCR results showed that the expression of UCA1 and PRL-3 was lower in the siRNA (si)-UCA1 and miR-495 mimic groups, with the expression of miR-495 exhibiting elevated levels compared with the control group (p < 0.05). We also found that the expressions of UCA1 and PRL-3 were significantly higher in the UCA1 group, whereas those in the miR-495 were lower (p < 0.05). We found no significant differences in UCA1, PRL-3, and miR-495 expression among the si-UCA1-NC, UCA1-NC, miR-495 mimic-NC, and UCA1 + miR-495 mimic groups (p > 0.05). This highlights how UCA1 was able to upregulate the expressions of PRL-3 by sponging miR-495 in GC cells (Figure 3I). The above results suggested that UCA1 upregulated the expression of PRL-3 by competitively binding to miR-495 in GC cells.

### Upregulated UCA1 and Downregulated miR-495 Promoted Cell Proliferation in GC

Cell Counting Kit-8 (CCK-8) assay (Figure 4) results revealed that cell proliferation in the si-UCA1-1 and si-UCA1-2 groups was inhibited 48 h after transfection compared with the si-UCA1-NC group (p < 0.05). Compared with the UCA1-NC group, cell proliferation in the UCA1 group was elevated (p < 0.05), and no significant differences in regard to cell proliferation in the UCA1 + miR-495 mimic group were observed (p > 0.05). Compared with the miR-495 mimic-NC group, the miR-495 mimic group showed inhibited cell proliferation. The above results suggested that the upregulation of UCA1 promoted cell proliferation, whereas the upregulation of miR-495 inhibited cell proliferation.

**Figure 4:** GC Cell Proliferation Was Facilitated by Upregulated UCA1 and Downregulated miR-495 *p < 0.05, versus the si-UCA1-NC group; ^#^p < 0.05, versus the UCA1-NC group; ^&^p < 0.05, versus the miR-495 mimic-NC group (measurement data at different time points were analyzed by repeated-measures ANOVA; each experiment was conducted three times independently).

### Upregulated UCA1 and Downregulated miR-495 Suppressed Cell Apoptosis in GC

Flow cytometry results (Figure 5) demonstrated that cell apoptosis was elevated in the si-UCA1-1 and si-UCA1-2 groups with increased cell numbers detected at the G0/G1 phase and decreased cell numbers detected at the S phase when compared with the si-UCA1-NC group. We found the mRNA and protein levels of Bcl-2 were decreased, whereas those of caspase-3 significantly increased (p < 0.05). Compared with the UCA1-NC group, the UCA1 group exhibited reduced cell apoptosis, accompanied by decreased cell numbers detected at the G0/G1 phase and increased cell numbers at the S phase, corresponding to increased mRNA and protein levels of Bcl-2 and decreased mRNA and protein levels of caspase-3 (p < 0.05). In addition, there was no significant change observed in the UCA1 + miR-495 mimic group (p > 0.05). Compared with the miR-495 mimic-NC group, the miR-495 mimic group showed increased cell apoptosis, increased cell numbers detected at the G0/G1 phase, and decreased cell numbers at the S phase, as well as decreased mRNA and protein levels of Bcl-2 and increased mRNA and protein levels of caspase-3 (p < 0.05). These findings suggested that the upregulation of UCA1 inhibits cell apoptosis, whereas the upregulation of miR-495 promotes cell apoptosis.

**Figure 5:** GC Cell Apoptosis Was Inhibited by Upregulated UCA1 and Downregulated miR-495 (A) Cell apoptosis in each group was detected by flow cytometry. (B) The apoptosis rate of cells in each group. (C) Cell cycle in each group detected by flow cytometry. (D) The cell-cycle distribution (%) of cells in each group. (E) The mRNA expression of Bcl-2 and caspase-3 detected by qRT-PCR. (F) The protein level of Bcl-2 and caspase-3 detected by western blot analysis. (G) Band patterns of Bcl-2 and caspase-3. *p < 0.05, versus the si-UCA1-NC group; ^#^p < 0.05, versus the UCA1-NC group; ^&^p < 0.05, versus the miR-495 mimic-NC group (measurement data were expressed as mean ± SD analyzed by independent sample t test; each experiment was conducted three times independently).

### Upregulated UCA1 and Downregulated miR-495 Promoted Cell Migration and Invasion in GC

Transwell assay (Figure 6) revealed that cell migration and invasion were reduced in the si-UCA1-1 and si-UCA1-2 groups, accompanied by decreased mRNA and protein levels of MMP-7 and MMP-2 when compared with the si-UCA1-NC group (p < 0.05). The UCA1 group, however, displayed enhanced migration and invasion abilities, accompanied by facilitated mRNA and protein levels of MMP-7 and MMP-2 as compared with the UCA1-NC group (p < 0.05). Moreover, there were no significant changes in the UCA1 + miR-495 mimic group (p > 0.05). Compared with the miR-495 mimic-NC group, the miR-495 mimic group showed inhibited cell migration and invasion abilities, as reflected by decreased mRNA and protein levels of MMP-7 and MMP-2 (p < 0.05). The above results suggested that upregulation of UCA1 promoted cell migration and invasion, whereas upregulation of miR-495 inhibited cell migration and invasion.

**Figure 6:** GC Cell Migration and Invasion Were Both Promoted by Upregulated UCA1 and Downregulated miR-495 (A) Cell migration detected by Transwell assay. (B) The number of migrating cells in each group. (C) Cell invasion detected by Transwell assay. (D) The number of invasive cells in each group. (E) The mRNA expression of MMP-7 and MMP-2 detected by qRT-PCR. (F) The protein level of MMP-7 and MMP-2 detected by western blot analysis. (G) Band patterns of MMP-7 and MMP-2. *p < 0.05, versus the si-UCA1-NC group; ^#^p < 0.05, versus the UCA1-NC group; ^&^p < 0.05, versus the miR-495 mimic-NC group (measurement data were expressed as mean ± SD and analyzed by independent sample t test; each experiment was conducted three times independently).

### Upregulated UCA1 and Downregulated miR-495 Promoted Peritoneal Metastasis of GC Cells in Nude Mice

As shown in Figure 7, compared with the control group, a decrease in the number of peritoneal metastasis nodules was detected in the si-UCA1 group and miR-495 mimic group, whereas an elevated number was observed in the UCA1 group (p < 0.05). However, no significant difference was found among the si-UCA1-NC group, UCA1-NC group, miR-495 mimic-NC group, and UCA1 + miR-495 mimic group (p > 0.05). These results demonstrated upregulation of UCA1 and downregulation of miR-495 can promote peritoneal metastasis of GC cell lines in nude mice.

**Figure 7:** Peritoneal Metastasis of GC Cells in Nude Mice Was Promoted by Upregulated UCA1 and Downregulated miR-495 (A) Peritoneal metastasis of GC cells in nude mice of each group. (B) The number of peritoneal tumor nodules in each group. The arrow indicates metastatic nodules; *p < 0.05, versus the control group (measurement data were expressed as mean ± SD and analyzed by one-way ANOVA; each experiment was conducted three times independently).

### Upregulated UCA1 and Downregulated miR-495 Promoted Gastric Tumor Formation in Nude Mice

The xenograft tumors were observed to evaluate tumor formation of GC cells in nude mice (Figure 8). When compared with the control group, suppressed tumor formation was observed in both the si-UCA1 and miR-495 mimic groups, whereas enhanced tumor formation was found in the UCA1 group (p < 0.05). No significant differences were observed in the si-UCA1-NC group, UCA1-NC group, miR-495 mimic-NC group, and UCA1 + miR-495 mimic group (p > 0.05). These results suggested that upregulation of UCA1 and downregulation of miR-495 promoted gastric tumor formation in nude mice.

**Figure 8:** Gastric Tumor Formation in Nude Mice Was Promoted by Upregulated UCA1 and Downregulated miR-495 (A) Representative tumors of nude mice in each group. (B) Tumor weight of mice in each group. (C) Tumor volume of mice in each group. *p < 0.05, versus the control group (the measurement data were expressed as mean ± SD and analyzed by one-way ANOVA; comparison of tumor volume at different time points was analyzed by repeated-measures of ANOVA; each experiment was conducted three times independently).

## Discussion

GC is the current fourth most commonly occurring cancer and the second leading cause of cancer deaths worldwide.^26^ Recent improvements in diagnostic tools have helped to facilitate early GC detection, which have gone a long way in increasing the chances of long-term survival in patients. However, the outcomes of GC patients suffering from advanced stages of the disease still remain poor. Therefore, a better understanding of the underlying mechanisms involved in GC may pave the way to novel therapies to combat the disease.

In this study, we examined the expression levels of UCA1 in both GC and normal gastric samples. Western blot assay and qRT-PCR techniques demonstrated that the expression of PRL-3 was increased in GC tissues and cells. Meanwhile, miRNA target prediction algorithms were applied to investigate the interaction between UCA1 and miR-495, as well as miR-495 and PRL-3, in GC, the results of which revealed that UCA1 upregulated the expression of PRL-3 by sponging miR-495. By studying the patterns of cell proliferation, apoptosis, migration, and invasion, we found that upregulated UCA1 and downregulated miR-495 could accelerate the progression of GC. Additionally, our *in vivo* experiments further verified our above findings. This study demonstrated that UCA1 promoted the proliferation, migration, and invasion of GC cells by sponging miR-495 to downregulate the expression of PRL-3.

Upregulation of UCA1 has been reported to play central roles in a variety of biological processes, including the proliferation and development of various tumors.^27^, ^28^, ^29^ A previous study demonstrated that UCA1 was highly expressed in GC and served as an oncogene in promoting cell proliferation in GC, whereas this particular lncRNA was found to be positively correlated with TNM staging in GC.^30^ Wang et al.^31^ demonstrated that UCA1 enhances GC cell metastasis by regulating the stability of GRK2 protein via promoting Cbl-c-mediated ubiquitination and degradation of GRK2, in addition to activating the extracellular signal-regulated kinase (ERK)-matrix metallopeptidase-9 (MMP-9) signaling pathway. UCA1 was also shown to promote epithelial-mesenchymal transition, which is known to be an essential early step in tumor metastasis,^32^ leading to overexpressed cyclin D1 and thus promoting cell-cycle progression in GC.^30^ Li et al. put forward a competing endogenous RNA hypothesis, which indicated how competition between lncRNAs, mRNAs, and pseudogene transcripts regulates each other’s expression by using miRNA response elements for the competitive binding of miRNAs, thereby emphasizing the importance of initiation and progression of malignancy.^17^

miRNAs regulate cellular activities by inhibiting related protein expression by base pairing with the 3′ UTR of the corresponding target mRNA.^19^ miRNAs have been shown to play pivotal roles in cancer initiation and progression because of their functions as either oncogenes or tumor suppressors.^33^^,^^34^ Various studies have demonstrated that miRNAs were correlated with the metastasis and prognosis of GC.^35^^,^^36^ The inhibition of GC cell migration and invasion by miR-495 was previously reported to function as a tumor suppressor by targeting the PRL-3 oncogene.^37^ Besides, miR-495 expression was found to be significantly downregulated in GC tissues and cells. The regulation of miR-495 levels can be explained by the extent of the methylation status by the miR-495 gene promoter or the regulation by transcription factors such as E12/E47, which are found in GC cells and breast cancer stem cells.^23^^,^^38^ Additionally, reports have suggested that miR-495 in SNU5 and SNU484 GC cells might possibly reduce cell proliferation, migration, and angiogenesis in the early phase of gastric tumorigenesis via regulating RUNX3 expression.^39^

Previous evidence has indicated that the expression of PRL-3 was significantly higher in primary GC with peritoneal metastasis compared with primary GC sites.^40^ Current literature has also highlighted that the expression of PRL-3 was associated with the extent of GC invasion and metastasis.^41^^,^^42^ PRL-3 is a tyrosine phosphatase that is required for the processes of tumor invasion, motility, and metastasis, which might be regulated by the dephosphorylation of several molecules including that of integrin, cadherin, and Ezrin.^6^ Zhang et al.^43^ reported that PRL-3 upregulated the expression of miR-210 in a hypoxia inducible factor 1 subunit alpha (HIF-1α) dependent manner under normoxia and hypoxia. They also demonstrated that PRL-3 also activated NF-κB signaling and promoted the expression of HIF-1α through modulating p65 phosphorylation, thereby contributing to migration and invasion of GC cells.^43^ At present, somewhat of a consensus exists suggesting that deregulated levels of PRL-3 expression share a strong correlation with cancer progression and poor survival, whereas postulations have been made highlighting its ability as a potential biomarker and therapeutic target in cancer.^44^

Collectively, the key findings in our study demonstrate that UCA1 upregulates the expression of PRL-3 through competitively binding to miR-495, which represents a mechanism by which the cell proliferation, invasion, and metastasis in GC were accelerated (Figure S1). We conclude that the UCA1/miR-495/PRL-3 axis underlines a potential therapeutic approach in the treatment of GC.

## Materials and Methods

### Ethics Statement

The study was conducted with the approval of the Animal Ethics Committee of The First Affiliated Hospital of Nanchang University. All participating patients were provided with information of the study and subsequently signed informed consent forms prior to enrolling in the study. All animal experiments were performed in accordance with the *Guide for the Care and Use of Laboratory Animals* published by the NIH.

### Bioinformatics Analysis

The GEO database (https://www.ncbi.nlm.nih.gov/geo) was used to retrieve GC-related microarray expression data (GEO: GSE103236 and GSE65801) and annotation probe files. The chips were obtained from the detection of Agilent-014850 Whole Human Genome Microarray 4x44K G4112F (Feature Number Version) and Agilent-028004 SurePrint G3 Human GE 8x60K Microarray (Probe Name Version). R software was used for background correction and normalization of each chip data.^45^ The linear model-empirical Bayes statistical method in the Limma installation package, combined with a traditional t test, was used for the nonspecific filtration of expression data, in order to screen the differentially expressed lncRNAs.^46^ The binding sites of gene and miRNAs were predicted by the databases microrna.org (http://www.microrna.org/microrna/getMirnaForm.do) and TargetScan (http://www.targetscan.org/vert_71/).

### Sample Collection

GC and normal adjacent tissues were obtained from 85 patients who were enrolled in this study. All patients were diagnosed with GC (stage I–IIIA) between June 2016 and August 2017. Every patient had undergone surgery at The First Affiliated Hospital of Nanchang University, with no local or systemic treatment received prior to surgery. The collected specimens were subsequently histologically evaluated along with the corresponding clinical data. All specimens were frozen in liquid nitrogen and stored at −80°C. The basic information of patients was collected, and the patients were asked to comply with follow-ups in order to record prognosis and clinical outcomes following treatment. The follow-up was started from the end of operation to December 2018 with a period of 3–30 months. Kaplan-Meier method with log rank test was used to analyze the relationship between UCA1 expression and GC patient survival.

### Cell Culture

Normal gastric epithelial cells (GSE-1) and five types of GC cells (MKN-28, MKN-45, SGC-7901, BGC-823, and MGC-803) were purchased from The Institute of Biochemistry and Cell Biology, Shanghai Institutes for Biological Sciences, Chinese Academy of Sciences (Shanghai, China). The cells were cultured in DMEM containing 10% fetal bovine serum, 1 × 10^5^ U/L penicillin, and 100 mg/L streptomycin in a humidified incubator at 37°C with 5% CO_2_. The culture medium was replaced every 2 days. Cell subculture was subsequently performed when cell confluence reached 80%–90% determined by visualization under a microscope. Cells at the logarithmic phase cells were selected for subsequent experiments. qRT-PCR was used to detect the expression levels of UCA1 in each cell line. Based on the obtained results, the cell lines with higher expressions of UCA1 were selected for subsequent experiments.

### Cell Transfection and Grouping

According to the sequences of UCA1 and miR-495 in NCBI, plasmids of si-UCA1, si-UCA1-NC, UCA1, UCA1-NC, miR-495 mimic, and miR-495 mimic-NC were designed by Sangon Biotech (Shanghai, China). Besides, the si-UCA1-1 and si-UCA1-2 groups were set to avoid the off-target effect. The cells at passage 3 were digested by trypsin and seeded into a 24-well plate, with the medium discarded for transfection. Cells were grouped according to transfection with different plasmids: control (BGC-823 cells without transfection), si-UCA1-1 (BGC-823 cells transfected with si-UCA1-1 plasmids), si-UCA1-2 (BGC-823 cells transfected with si-UCA1-2 plasmids), si-UCA1-NC (BGC-823 cells transfected with si-UCA1-NC plasmids), UCA1 (BGC-823 cells transfected with UCA1 plasmids), UCA1-NC (BGC-823 cells transfected with UCA1-NC plasmids), miR-495 mimic (BGC-823 cells transfected with miR-495 mimic plasmids), miR-495 mimic-NC (BGC-823 cells transfected with miR-495 mimic-NC plasmids), and UCA1 + miR-495 mimic (BGC-823 cells transfected with UCA1 plasmids and miR-495 mimic plasmids).

Cell transfection was performed using Lipofectamine 2000 (Invitrogen, USA), in strict accordance with the instructions provided by the kit. BGC-823 cells were seeded into six-well plates with a density of 2 × 10^5^ cells/well. After cell adherence, the cells were cultured in a penicillin/streptomycin free medium for 12 h prior to transfection. Then 100 pmol plasmids were diluted with 250 μL serum-free Opti-MEM and incubated at room temperature for 5 min. During incubation, 4 μL Lipofectamine 2000 was diluted with 250 μL serum-free Opti-MEM. The plasmids and Lipofectamine 2000 were then mixed, incubated for 20 min at room temperature, and placed into the plates containing 250 μL of OPTI-MEM. A culture was then conducted at 37°C conditions with 5% CO_2_, with the previous culture medium replaced by a complete medium after 6 h had passed. In order to select well-transfected cells, the cells were cultured in G418 (1,000–2,000 μg/mL) for 4 weeks, and 48 h after transfection the medium was replaced at 3- to 5-d intervals.

### qRT-PCR

The TRIzol Reagent (Takara Biotechnology, China) was used to extract the total RNA from each group. NanoDrop ND-1000 (NanoDrop Technologies, USA) was used to measure RNA purity and concentration from each sample. Reverse transcription was performed using a PrimeScript RT reagent Kit (Takara Biotechnology, China). DNA concentration and purity were detected using a UV spectrophotometer and 1% agarose gel (A260/A280 > 1.8). The U6 gene was used as the internal reference for UCA1 and miR-495 using the Quanti-Tect SYBR Green PCR kit as the qRT-PCR reagent. GAPDH gene was the internal reference for the other genes that utilizes SYBR Premix Ex TaqII Kit (Takara, Japan) as the qRT-PCR reagent. The primers used in this study are illustrated in Table S2. All experiments were conducted using the ABI7500 qPCR instrument (Applied Biosystems, USA). The 2^−ΔΔCT^ method was used to calculate the relative expression levels of the target genes.

### Western Blot Analysis

The cells were collected for protein extraction 72 h after transfection. Total protein was extracted using a Radioimmunoprecipitation assay buffer containing a protease inhibitor. Protein concentration was determined using a bicinchoninic acid (BCA) Protein Assay Kit (Pierce, USA). A 30-μg loading sample was then added to each well, mixed with loading buffer, boiled for 5 min, incubated in an ice bath, centrifuged, and separated using 12.5% polyacrylamide gel electrophoresis. Separated proteins were transferred onto a polyvinylidene fluoride membrane. The membrane was blocked with 5% skimmed milk powder for 1 h and incubated with the following antibodies: rabbit anti-human PRL-3 (1:300, P0498; Sigma-Aldrich Chemical Company, USA), Bcl-2 (1:1,000, ab32124; Abcam, USA), caspase-3 (9661; Cell Signaling Technologies [CST], USA), MMP-7 (1:1,000, ab207299; Abcam, USA), and MMP-2 (1:500–2,000, ab37150; Abcam, USA) at 4°C overnight. On the following day, the membrane was rinsed three times with PBS, 5 min each time, and incubated with HRP-labeled goat anti-rabbit IgG antibody (1:2,000–20,000, ab6721; Abcam, Cambridge, MA, USA) at 37°C for 1 h, followed by PBS rinse. Enhanced chemiluminescence (Pierce, USA) was used to visualize the protein bands for 1 min. GAPDH served as the internal reference. The ratio of the gray value of target bands to that of GAPDH was analyzed in order to calculate the relative expression of the target genes.

### RNA FISH

In order to separate the plasma and nucleus, the cells were initially digested using trypsin (centrifugation for 5 min) and then washed with cold PBS. The cells were then transferred into a 1.5-mL eppendorf tube followed by centrifugation for 2 min. The precipitate was mixed with pre-cooled cytoplasmic protein extraction reagent (CER) I using vortex at maximum speed for 15 s. Cells were lysed on ice for 10 min, vortexed with pre-cooled CER II, placed on ice for 1 min, and centrifuged at 4°C for 5 min. The supernatant consisting of cytoplasmic components was extracted and then preserved at −80°C. Afterward, the cells were washed three times with PBS, vortexed with pre-cooled NER for 15 s, placed on ice for 10 min, and vortexed again for 15 s. After centrifugation for 10 min at 4°C, the supernatant consisting of nuclear components was obtained and preserved at −80°C.

The FISH procedure was performed according to the following protocol: on the first day, sections were dried at 50°C for 15–30 min, fixed in diethyl pyrocarbonate (DEPC)-4% paraformaldehyde (PFA) at room temperature for 20 min, rinsed with 1× DEPC-PBS A, rinsed with 1 × DEPC-PBS B for 5 min, followed by Proteinase K treatment at room temperature for 10 min. The sections were rewashed in 1× DEPC-PBS B, fixed in DEPC-4% PFA for 10 min, rinsed in 1× DEPC-PBS A, and immersed in 1× DEPC-PBS B for 5 min. After that, sections were treated with acetic acid by incubation with 0.1 M RNase-free Triethanolamine at room temperature for 10 min, followed by rinsing with 1× DEPC-PBS B and immersion in 1× DEPC-PBS C for 5 min. Next, 200 μL of pre-hybrids was added to each section and left to incubate in a hybrid box for 1 h at room temperature. Next, 0.1–0.2 ng/μL RNA probe was denatured for 5 min at 85°C and then immediately cooled on ice, with each section incubated using an RNA probe at 65°C for 14 h. On the second day, preheated 0.2× saline sodium citrate (SSC) A, B, and C were used three times to immerse sections 20 min each time. 0.2× SSC D was used for immersion for 5 min, buffer B 1 solution was used for immersion at room temperature twice (5 min each time), buffer B 2 solution was used for blocking at room temperature for 1 h, and buffer B 2 diluted with anti-DIG-AP Fab antibody (1:5,000) was added for incubation at 4°C overnight. On the third day, the slices were immersed in buffer B 1 three times at room temperature, 20 min each time, balanced twice with buffer B 3, 5–10 min each time, and mixed with fresh 5-bromo-4-chloro-3-indolyl phosphate/Nitroblue tetrazolium chloride liquid for 3–24 h in the dark. The reaction was stopped and terminated with double-distilled H_2_O (ddH_2_O).

### Bioinformatics Prediction and Dual-Luc Reporter Gene Assay

The biological prediction website was used to predict the targeting relationship between UCA1 and miR-495 and that between miR-495 and PRL-3. The primers of UCA1-WT and -Mut type were synthesized by Sangon Biotech (Shanghai), and dual-Luc reporter gene assay was conducted to determine the targeting relationship between UCA1 and miR-495. Double-enzyme digestion was performed using HindIII and BglII restriction sites. PCR was then used to amplify the DNA sequence. The large fragments were collected after the pGL3-Basic Luc reporter had been subjected to enzyme digestion with restriction endonuclease HindIII and BglII. UCA1-WT-Luc and UCA1-Mut-Luc were obtained by digesting the plasmids using Ligase 4. After vector transformation into *Escherichia coli* and identification by PCR, the colony-containing target fragments were used for plasmid extraction and sequencing. The 293T cells were subsequently divided into four groups: group A, cells transfected with UCA1-WT-Luc plasmid and miR-495 mimic plasmid; group B, cells transfected with UCA1-WT-Luc plasmid and miR-495 mimic-NC plasmid; group C, cells transfected with UCA1-Mut-Luc plasmid and miR-495 mimic plasmid; and group D, cells transfected with UCA1-Mut-Lu plasmid and miR-495 mimic-NC plasmid. Cell transfection was conducted with Lipofectamine 2000 (Invitrogen, USA), and procedures were carried out in accordance with the instructions provided by the kit. The medium was changed at the 6-h point after transfection, and the cells were collected 24 h later, followed by detection of Luc activity using the Dual-Luc Reporter Assay Kit (Promega, USA) and enzyme labeling instrument at 560 nm (MK3; Thermo, USA).

WT PRL-3 fluorescein reporter plasmid (PRL-3-WT-Luc) containing WT PRL-3 sequence and Mut PRL-3 fluorescein reporter plasmid (PRL-3-Mut-Luc) containing Mut PRL-3 sequence were purchased from Shanghai Genechem (China). 293T cells were divided into four groups: group A, cells transfected with PRL-3-WT-Luc plasmid and miR-495 mimic plasmid; group B, cells transfected with PRL-3-WT-Luc plasmid and miR-495 mimic-NC plasmid; group C, cells transfected with PRL-3-Mut-Luc plasmid and miR-495 mimic plasmid; and group D, cells transfected with PRL-3-Mut-Lu plasmid and miR-495 mimic-NC plasmid. The following steps were conducted in the same manner as the aforementioned procedures. The experiments were repeated three times.

### RNA Pull-Down

The total RNA was transcribed using an AmpliScribe T7-Flash Biotin-RNA Transcription Kit (Epicenter, China). RNA was purified by RNeasy Plus Mini Kit transcription and DNase I (QIAGEN, Germany), and labeled with biotin by Biotin RNA Labeling Mix (Ambio Life, USA). The labeled RNA was then added with the RNA structure buffer (10 mM Tris [pH 7.0], 0.1M KCl, and 10 mM MgCl_2_) and left to react at 90°C for 2 min. RNA was then incubated on ice for 20 min and left at room temperature for 20 min. Afterward, RNA and protein products were mixed together and left to incubate at room temperature for 1 h. This was followed by the addition of Streptavidin magnetic beads (GE Healthcare) at room temperature for 1 h and a rinse with ddH_2_O in preparation for the next experiment.

### RIP

Cell lysis solution (Sigma-Aldrich Chemical Company, USA) was added to 3 μg of cells and left to incubate at 4°C for 1 h. Cells were centrifuged at 12,000 × *g* at 4°C for 10 min in order to collect the supernatant, which was then transferred into RNase-free tubes. After that, the tubes were mixed with 400 ng of labeled RNA and 500 μL of RIP buffer (Millipore, USA), and allowed to mix for 1 h, followed by the addition of 50 μL of Streptavidin agarose beads (Invitrogen, USA) for 1 h, followed by five RIP washes. The washing liquid was used for qRT-PCR, and samples were added with 5 × *g* loading buffer, followed by incubation at 95°C for 5 min and western blot analysis. These experiments were repeated three times.

### CCK-8 Assay

At 48 h after transfection, cells in the logarithmic growth phase were collected and used to prepare a suspension with a concentration of 1 × 10^4^ cells/mL in DMEM containing 10% fetal bovine serum culture and inoculated into 96-well plates. According to individual cell grouping, each group was prepared with eight wells, 100 μL in each well. The cells were then cultured in a cell incubator with 5% CO_2_ at 37°C. After each time interval of 24, 48, and 72 h, 10 μL of CCK-8 (Sigma-Aldrich Chemical Company, USA) was added into each well and allowed to culture for an additional 2 h. The optical density (OD) values at 450 nm were recorded from each of the samples using a microplate reader (NYW-96M; NYAW, China). The experiments were repeated three times.

### Flow Cytometry

After cell transfection for 48 h, the cells were digested with 0.25% trypsin and adjusted to obtain a cell concentration to 1 × 10^6^ cells/mL. Then 1 mL of the cells was centrifuged at 1,500 rpm for 10 min. The cells were then washed with 2 mL of PBS and re-centrifuged again. The sediment was added to the precooled 70% ethanol for fixing at 4°C overnight, followed by two PBS washes on the following day. Afterward, 100 μL of cell suspension was added to 50 μg of propidium iodide (PI) containing RNase (Qcbio Science & Technologies, China) and left to react for 30 min in the dark. Cell-cycle patterns were recorded at 488 nm using a flow cytometer (BD, USA).

Cell apoptosis was detected by Annexin V-fluorescein isothiocyanate (FITC)/PI double staining. After culturing at 37°C with 5% CO_2_ for 48 h, the cells were washed twice with PBS, centrifuged, resuspended in 200 μL of binding buffer, and stained with 10 μL of Annexin V-FITC (ab14085; Abcam, USA) and 5 μL PI successively for 15 min in the dark. Next, 300 μL of binding buffer was then added, and cell apoptosis was detected at 488 nm using a flow cytometer. The experiments were repeated three times.

### Transwell Assay

At 24 h after transfection, cells were digested with trypsin and suspended in a serum-free medium containing BSA to prepare a cell suspension. Then 200 μL of cell suspension was added to an 8-mm Transwell chamber (Transwell, UK) filled with a 24-well plate. Subsequently, 500 μL medium containing 20% FBS was added into the lower chamber of the 24-well plate for incubation at 37°C with 5% CO_2_ for 24–48 h. Cotton swabs were used to wipe cells in the upper chamber, followed by rinse with PBS three to five times. Cells were then fixed with methanol for 20 min, stained with 0.1% crystal violet for 30 min at 37°C, and rewashed with PBS to remove the superfluous crystal violet. Afterward, cells were immersed in 33% glacial acetic acid and left to oscillate for 10 min. Cell migration and invasion were detected by a microplate reader (Tecan, China) at 570 nm. Cell invasion experimental procedures were carried out according to the same as those that were mentioned in previous experiments with the exception of the Transwell chamber, which was instead added with 50 mg/L Matrigel (dilution of 1:8; Millipore, USA). The experiments were repeated three times.

### Peritoneal Metastasis in Nude Mice

The male 5-week-old BALB/c nude mice were employed for the following experiment, with 12 mice in each group. Each mouse had free access to food and water in 50%–60% humidity with adequate ventilation, normal room temperature, with alternating light and dark cycles. Six nude mice for each group were used for peritoneal metastasis experiment. At 24 h after transfection, cells were treated with trypsin, washed twice with PBS, and resuspended in serum-free medium 1640 to adjust the cell concentration to 5 × 10^6^ cells/mL. Afterward, 1 mL of cell suspension was injected into the peritoneal cavity of each nude mouse. After 21 d, six nude mice were executed, and the number of peritoneal tumor nodules was counted and recorded. The remaining nude mice were raised continually for 120 d, in order to observe tumor progression.

### Cellular Tumorigenicity in Nude Mice

Six nude mice in each group were used for tumor formation experiment. Each mouse was allowed free access to food and water consumption in conditions of 50%–60% humidity, good ventilation, normal room temperature, and alternating light/dark cycles. At 24 h after transfection, the cells were digested with trypsin, washed twice with PBS, and resuspended in serum-free medium 1640 for cell counting. Next, 5 × 10^6^ cells were suspended in 0.1 mL serum-free DMEM, mixed with 0.1 mL Extracellularmatrix gel, and injected into the peritoneal cavity of nude mice. The same number of cells was then injected into the same site of mice after 3 days. Tumor formation was observed at 6-day intervals after initial injection. The sizes of the tumor were measured and recorded each time. Four weeks after tumor formation, the nude mice were executed for sample collection to measure the weight and size of the specimen. The calculation formula applied was (L × W^2^)/2, in which L represented the length of the tumor, and W was the width of the tumor.

### Statistical Analysis

All data were analyzed by SPSS 21.0 software (IBM, Armonk, NY, USA). The measurement data were expressed as mean ± SD. Count data were expressed as number of cases and percentages. Comparisons between two groups were made using a paired t test for normally distributed measurement data and non-parametric Wilcoxon rank sum for skewed data. Comparisons of measurement data among multiple groups were analyzed by one-way ANOVA. Multiple comparisons of the average value of samples were analyzed by the least significant difference (LSD). Cell viability at different time points was analyzed by repeated-measures ANOVA. A p value <0.05 was indicative of statistical significance.

## Author Contributions

Y.C. and G.-Y.Z. designed the study. J.-B.X. and Y.L. collated the data, carried out data analyses, and produced the initial draft of the manuscript. Z.-G.J. and Z.-R.L. contributed to drafting and polishing the manuscript. All authors have read and approved the final submitted manuscript.

## Conflicts of Interest

The authors declare no competing interests.

## Supplemental Information

Document S1. Figure S1 and Tables S1 and S2

Document S2. Article plus Supplemental Information
